RETRACTED

# Efficacy of Oxidized Regenerated Cellulose/Collagen Dressing for Management of Skin Wounds: A Systematic Review and Meta-Analysis

**DOI:** 10.1155/2021/1058671

**Published:** 2021-08-04

**Authors:** Li Zhang, Simei Wang, Meihua Tan, Hongwei Zhou, Ying Tang, Yan Zou

**Affiliations:** ^1^Department of Orthopedics and Trauma, The Affifiliated Nanhua Hospital, University of South China, Hengyang, Hunan, China; ^2^Department of Wound Stoma Care, The Affifiliated Nanhua Hospital, University of South China, Hengyang, Hunan, China; ^3^Department of Hand and Foot Surgery, The Affifiliated Nanhua Hospital, University of South China, Hengyang, Hunan, China

## Abstract

**Objective:**

The purpose of this study was to evaluate the wound healing efficacy of oxidized regenerated cellulose (ORC)/collagen dressing and ORC/collagen/silver-ORC dressings compared to standard of care or control in treatment of chronic skin wounds such as diabetic foot ulcers (DFUs), venous leg ulcers (VLUs), and pressure injuries sore ulcers (PISUs).

**Methods:**

An electronic search was carried out in four popular databases PubMed, Scopus, Embase, and CENTRAL to identify thirteen included studies, comparing the clinical efficacy of ORC/collagen dressings when compared to control in management of chronic skin wounds, especially DFUs, VLUs, and PISUs, and skin graft donor site wounds.

**Results:**

Consolidated data from thirteen comparative clinical studies undertaken for management of DFUs, VLUs, and PISUs showed favorable outcomes towards use of ORC/collagen compared to other traditional and hydrocolloid foam dressings in terms of wound healing rate (*P*=0.02) and percentage wound relative reduction (*P*=0.003). The time taken to achieve complete wound healing in the included studies did not show any statistical significant difference (*P*=0.24). There was no significant difference in adverse events between ORC/collagen-treated group and comparative group (*P*=0.19).

**Conclusion:**

ORC/collagen wound dressings are beneficial in terms of improved wound healing rate and percentage wound relative reduction compared to already existing traditional standard of care with non-MMP, inhibiting biomaterials such as moistened gauze, autologous growth factors, hydrocolloid foam dressings, or ovine extracellular matrix.

## 1. Introduction

Wound is defined as a disruption in cutaneous structure and function, potentially involving underlying soft tissue [1]. Various factors that can result in impaired wound healing include aging, malnutrition, diabetes, vascular disease, and immunosuppression [2]. Chronic skin wounds occur when normal wound healing is dysregulated, resulting in a delay or arrest in one of the stages of wound healing. Prolongation of the inflammatory phase is the most common cause, usually due to wound infection or chronic irritation. Other possible mechanisms are tissue and wound hypoxia or failed epithelialization [3]. Surgeons sometimes reexcise the tissue and convert the chronic wound back into an acute one for faster healing and tissue regeneration [4]. The ultimate requirement for complete wound healing involves proper nursing of wound by application of wound dressings or wound care products [5]. The wound dressings used in management of chronic wounds needs to be cost-effective and clinically efficient, high patient acceptance, and most importantly improved patient's quality of life [6].

RETRACTED

Conventional wound dressings used for wound care management include traditional moistened gauze or petrolatum and modern dressings including alginates, hydrofibers, hydrogels, films, and biological agents including ovine collagen [7]. However, these dressings are permeable to bacteria and not conducive for creating a physiological environment. Nowadays, use of biological dressings like collagen is impermeable to bacteria, thereby reducing colonization. The popularity of collagen dressing nowadays ought to its ease of application and being natural, nonimmunogenic, nonpyrogenic, hypoallergenic, and pain-free healing [7]. Autologous platelet concentrates [8, 9] also have been beneficial and cost-effective in promoting wound healing.

Chronic wounds often present with elevated levels of matrix metalloproteinases (MMPs), which carryout proteolysis and inactivate the intrinsic growth factors involved in wound healing [10]. This may be the reason for which chronic skin wound takes longer time to heal [11]. The collagen dressings are found to inhibit the action of MMPs and encourage speedy deposition and proper organization of freshly formed collagen fibrils and granulation tissue formation, forming a bed to promote wound healing. These collagen fibrils undergo maturation and aid in epithelial migration from wound periphery for complete wound closure [12].

Oxidized regenerated cellulose (ORC)/collagen matrix is one such MMP inhibiting biomaterial which intensifies the wound healing environment by binding and inactivating excess levels of proteases and gelatinases in wound exudates [13]. Wu et al. [14] showed a statistical significant decrease in elastase, plasmin, and gelastinase activity in patients with venous leg ulcers (VLUs) treated with ORC/collagen matrix and also showed a significant and immediate reduction in protease activity in wound exudates from VLUs. Motzkau et al. in 2011 demonstrated the effects of MMP activity in the exudate of chronic diabetic foot ulcers (DFUs) treated with ORC/collagen dressing and found significantly decreased MMP-2 levels on day 5 of treatment [15].

RETRACTED

Several studies have also assessed the efficacy of ORC/collagen dressing and ORC/collagen/silver-ORC dressings for wound management [16, 17]. However, to the best of our knowledge, no meta-analysis has been conducted till date proving the efficacy of ORC/collagen in different chronic skin wounds. Therefore, the purpose of this study was to evaluate the wound healing efficacy of ORC/collagen dressing and ORC/collagen/silver-ORC dressings compared to standard of care or control in the treatment of chronic skin wounds.

## 2. Methods

This systematic review and meta-analysis was carried out with strict adherence to preferred reporting items for systematic review and meta-analysis (PRISMA) guidelines [18]. A prior protocol was framed to facilitate the smooth conduct in performing this systematic review.

### 2.1. Research Question

What is the wound healing efficacy of ORC/collagen dressing and ORC/collagen/silver-ORC dressings compared to standard of care or control in the treatment of chronic skin wounds? Patient or population (P): participants with chronic skin wounds (DFUs, VLUs, PIs, etc.); intervention (I): wound dressing with ORC/collagen or ORC/collagen/silver-ORC dressings; comparison (C): standard of wound care or control; outcome (O): wound healing rate, wound reduction, time taken for complete healing, adverse events, etc.

### 2.2. Search Strategy

An electronic search was carried out in four popular databases PubMed, Scopus, Embase, and CENTRAL to identify potential eligible studies. The keywords used for the search strategy include collagen, oxidized regenerated cellulose, collagen/ORC wound dressing, wound healing, chronic skin wounds, diabetic foot ulcer, venous leg ulcer, and pressure injuries. The keywords were combined in the advanced search using Boolean operators. Additionally, a manual search was also performed in published issues of Advances in Skin and Wound Care, Journal of Wound Care, International Wound Journal, Wounds, and International Journal of Lower Extremity Wounds. The bibliography section of the potentially eligible studies and previously performed systematic reviews was also inspected for any relevant studies. No restriction in publication year and language was applied. The search results from different electronic databases and manual search were imported to a citation manager (endnote) to remove duplicates and subsequently subjected to assessment for study selection.

### 2.3. Study Selection

The retrieved studies were subjected to title and abstract screening by two independent reviewers based on relevancy. The relevant articles were then assessed by retrieving full text for each of the potentially eligible studies. The criteria for inclusion of studies are as follows:

1. Comparative clinical studies
2. Application of ORC/collagen or ORC/collagen/silver-ORC dressings compared to control in management of chronic skin wounds (DFUs, VLUs, PIs, etc.)
3. Studies with minimum sample size of 10 (5 per group)

The case reports, case series, cohort studies, and clinical studies assessing another MMP inhibiting dressing with ORC/collagen dressing were excluded. The reasons of exclusion of the eligible studies were also provided. Any disagreement between the two reviewers with regard to study selection and exclusion was resolved by consensus with a third reviewer.

RETRACTED

### 2.4. Data Extraction

The data extraction from the included trials was carried out by two independent reviewers using an excel spreadsheet. The demographic data of participants such as age, gender, type and duration of wound, and wound area and size; interventional characteristics such as type of wound dressing, change of dressing per week, and follow-up; and outcome variables such as wound closure, percentage of wound relative reduction, time taken for complete epithelialization and granulation bed formation, and adverse events were recorded for each included trial. In case of any missing or unclear data, the authors were contacted via e-mail to seek out clarifications.

### 2.5. Data Synthesis

The data extracted from the included trials were subjected to both qualitative and quantitative analysis. The demographic data and interventional characteristics along with certain outcomes with little similarities were qualitatively analyzed and tabulated for better representation. The qualitative analyses of the similar outcome assessment were carried out using meta-analysis. The meta-analysis was performed by using RevMan 5.3v. The heterogeneity among the studies was calculated using i2 statistics. A random or fixed effect model for meta-analysis was employed based on the i2 value. i2 of less than 40% was considered unimportant while that of more than 40% was viewed as moderate to considerable heterogeneity.

### 2.6. Risk of Bias Assessment

The risk of bias analysis was carried out using Cochrane risk of bias tool [19] by two independent reviewers. The included trials were analyzed for bias in selection of participants by evaluating randomization process and allocation concealment methods; bias in blinding of participants and personnel; bias in blinding of outcome assessors; and bias in selective reporting of results and lost to follow-up. The studies were graded as low, moderate, and high risk based on adequacy of the abovementioned domains.

RETRACTED

## 3. Results

### 3.1. Search Results

This systematic review assessed the data from 13 included studies [13, 15, 20–30] comparing the clinical efficacy of ORC/collagen dressings when compared to control in the management of chronic skin wounds, especially DFUs, VLUs, and PIs. The electronic search was carried out in all 4 databases and the manual search retrieved 699 articles, where the total studies identified were 545 after removal of duplicates. After careful title and abstract screening, only eighteen studies were found potentially eligible and relevant. Full text evaluations of eighteen studies were carried out to find only thirteen studies satisfying the inclusion criteria. The rest of the five studies were excluded and detailed reasons of exclusion were provided. The study selection and exclusion process is depicted in Figure 1.

### 3.2. Demographic and Interventional Characteristics

There were 10 randomized clinical trials [13, 15, 21, 22, 24–27, 29, 30], 2 comparative clinical trials [23, 28], and 1 comparative retrospective study [20], comparing the use of ORC/collagen dressings and other wound dressings as control. 8 included studies [15, 22–24, 26–29] assessed the effect of ORC/collagen on healing of DFUs, 2 studies [13, 21] evaluated healing of VLUs, 1 study [25] evaluated healing of PIs, and another study assessed healing of skin graft donor site wounds. A consolidated total of 1538 wounds were evaluated in 13 included studies [13, 15, 20–30]. Out of which, 782 wounds were treated with ORC/collagen dressing and rest of 736 wounds were treated either with standard wound care, moistened gauze, hydrocolloid foam, or ovine-based extracellular matrix. The age range of the patients presented with chronic skin wounds is from 18 to 88 years. The demographic data from all included studies is provided in Table 1. The interventional characteristics from all included studies are provided in Table 2. The details of the type, duration, area of wound, the times of dressing change in every week, and the follow‐up duration were recorded in the individual files. The follow-up duration among the included studies ranged from a minimum follow-up period of 5 days and maximum follow-up period of up to 16 weeks.

### 3.3. Meta-Analysis

The quantitative analysis for the outcomes was carried out by meta-analyzing the data only if more than 2 similar studies were found to report a similar outcome with a common unit of measurement. The meta-analysis was performed for the following parameters.

#### 3.3.1. Wound Healing Rate

Six studies [21–23, 27, 29, 30] were analyzed to compare the wound healing rate between the ORC/collagen group and control group. The overall OR 1.79 [1.09, 2.94] was found to be significantly favoring ORC/collagen-treated group (*P*=0.02). The heterogeneity among the studies was found to be moderate (*i*2 = 57%), as shown in Figure 2.

RETRACTED

#### 3.3.2. Time to Achieve Complete Wound Healing

Only three studies [27, 29, 30] were analyzed to compare the time to achieve complete wound healing between the ORC/collagen group and control group. The overall MD −2.25 [−22.95, 18.46] between both groups was found nonsignificant (*P*=0.83). The heterogeneity among the studies was also found to be high (*i*2 = 97%), as shown in Figure 3.

#### 3.3.3. Percentage Wound Relative Reduction

Only three studies [21, 25, 28] were analyzed to compare the percentage wound relative reduction between the ORC/collagen group and control group. The overall MD 18.15 [6.09, 30.21] was found to be significantly favoring ORC/collagen-treated group (*P*=0.003). The heterogeneity among the studies was also found to be low (*i*2 = 29%), as shown in Figure 4.

#### 3.3.4. Adverse Events in Wound Healing

Four studies [21, 22, 29, 30] were analyzed to compare the adverse events in wound healing between the ORC/collagen group and control group. The overall RD −0.08 [−0.21, 0.04] between both groups was found nonsignificant (*P*=0.19). The heterogeneity among the studies was also found to be moderate (*i*2 = 54%), as shown in Figure 5.

### 3.4. Risk of Bias Assessment

The included studies were assessed to have low to moderate risk of bias, except 2 studies [15, 23], which were assessed as high risk due to lack in randomization and blinding of outcome assessor, respectively, as shown in Figure 6.

## 4. Discussion

This systematic review aimed at evaluating the wound healing efficacy and adverse events associated with ORC/collagen dressings in treatment of various chronic skin wounds. Consolidated data from thirteen comparative clinical studies undertaken for management of DFUs, VLUs, and PIs showed favorable outcomes towards use of ORC/collagen compared to other traditional and hydrocolloid foam dressings in terms of wound healing rate and percentage wound relative reduction. The time taken to achieve complete wound healing in the included studies did not show any statistical significant difference. There was no significant difference in adverse events between ORC/collagen-treated group and comparative group (*P*=0.19).

The beneficial effect of ORC/collagen can be due to its ability to absorb oxygen free radicals, bind excess iron, and protect growth factors present in chronic wound fluid [31]. The above mechanism may explain how ORC/collagen can redress the imbalance of the chronic wound environment and therefore may have a beneficial effect in the treatment of chronic skin wounds.

RETRACTED

It is proven that there exists a complex intrinsic interaction between cells and its mediators in response to tissue injury. Wounds that do not progress beyond the inflammatory phase often demonstrate an increased activity of proteases such as MMPs and elastase, as well as the persistence of inflammatory cells [32]. There is also a downregulation of tissue inhibitor of matrix metalloproteinase activity. In particular, the inflammatory response seems to be high in chronic skin wounds, characterized by increased levels of proinflammatory cytokines and proteases [33]. While controlling levels of inflammation and protease expression is a critical part of normal wound healing, elevated and prolonged expression of proteases produced during the inflammatory phase of healing can lead to excessive ECM degradation associated with impaired healing [11]. Therefore, use of a collagen-based MMP inhibiting biomaterial as wound dressing has been popular nowadays.

The protease inhibitory role of ORC/collagen is well established in many in vitro and in vivo studies. Smeets et al. in 2008 [13] showed that the patients treated with ORC/collagen matrix showed a significant decrease in elastase, plasmin, and gelatinase activity as compared with the control group, with no significant difference in the MMP-2 concentrations between the two groups. However, the results showed a significant and immediate reduction in protease activity in wound exudates from VLUs treated with ORC/collagen.

Apart from this, ORC/collagen was also found to promote fibroblast migration and proliferation in vitro [34]. The in vivo effects of ORC/collagen on wound of diabetic mice were also investigated in terms of wound closure and histological analysis and concluded that the ORC/collagen accelerated wound closure and histological appearance by promoting fibroblastic activity and thereby supporting complete epithelialization [34]. This could be a reason which could explain our favorable results towards ORC/collagen dressing in terms of faster wound healing rate and improved percentage wound relative reduction. However, no significant difference was noted in the time to complete wound closure between ORC/collagen and comparative dressings. Indeed, complete wound healing does not often require just one dressing and at the reepithelialization stage or when exudate disappears, the dressing needs to be discontinued. This is an important reason for the nonsignificant difference between the two groups of our review.

Many of the included studies [13, 15, 24–26] in this review estimated the protease, elastase, and other MMP levels in the wound exudates and compared between the ORC/collagen-treated wounds and other traditional or biologically dressed wounds. The comparison of anti-MMP activity of ORC/collagen was however out of the scope of this review. Our review only analyzed the wound healing efficacy and, to certain level, the safety profile of using ORC/collagen over other controls.

RETRACTED

It was also noted that the patients treated with ORC/collagen required less changes in dressing per week per patient. However, a quantitative analysis could not be performed due to lack of similar data representation. There was no significant difference observed in adverse events or complications associated with ORC/collagen dressings compared to controls. The adverse events associated with the dressing included infections, septicemia, and failure in granulation bed formation. The extent of adverse events observed with use of ORC/collagen and silver-ORC/collagen was similar to that of the materials used as controls for wound healing.

The moderate to high heterogeneity among the studies analyzing time to achieve complete healing, healing rate, and adverse events could be explained by the fact that there had been variation in systemic status of the patients, wound size and duration, and follow-up period. The diabetic foot ulcers are difficult to heal compared to other chronic skin wounds due to intrinsic impairment of wound healing response [35]. The limitation of this review includes difficultly in conducting subgroup analysis based on type of wounds (DFUs, VLUs, PIs, etc.) and between silver-ORC and ORC/collagen dressing, due to lack of sufficient studies.

## 5. Conclusions

ORC/collagen wound dressings are beneficial in terms of improved wound healing rate and percentage wound relative reduction compared to already existing traditional standard of care with non-MMP, inhibiting biomaterials such as traditional moistened gauze or petrolatum and modern dressings including foams, alginates, hydrofibers, hydrogels, hydrocolloids, films, and biological agents such as ovine collagen. Future comparative studies of high quality evidence are required to further establish the beneficial and protective effect of ORC/collagen dressings in the treatment of chronic skin wounds.

## Figures and Tables

**Figure 1:** PRISMA flow chart showing study selection process.

**Figure 2:** Forest plot showing comparison of complete wound healing rate between ORC/collagen and control groups.

**Figure 3:** Forest plot showing comparison of time taken to achieve complete wound healing between ORC/collagen and control groups.

**Figure 4:** Forest plot showing comparison of percentage wound relative reduction between ORC/collagen and control groups.

RETRACTED

**Figure 5:** Forest plot showing comparison of adverse events in wound healing between ORC/collagen and control groups.

**Figure 6:** Risk of (a) bias summary and (b) bias graph of all included studies.

**Table 1:** Demographic data of all included studies.

Authors	Study design	Centres	No. of patients	Age	Gender (M/F)	Test dressing	Control dressing	Type of wound
Veves et al., 2002 [29]	RCT	11	276	58.3 (23–85)	203/73	ORC/collagen matrix	Gauze	DFUs
Vin et al., 2002 [30]	RCT	14	73	33–88	26/47	ORC/collagen matrix	Nonadherent dressing (Adaptic)	VLUs
Lobmann et al., 2006 [26]	RCT	1	33	64 ± 11	NR	ORC/collagen matrix	Good standard wound care	DFUs
Luis Lazaro-Martinez et al., 2007 [27]	RCT	1	40	NR	NR	ORC/collagen matrix	Hydroactive dressing	DFUs
Kakagia et al., 2007 [24]	RCT	1	54	NR	22/29	ORC/collagen matrix	Autologous growth factors	DFUs
Smeets et al., 2008 [13]	RCT	NR	27	63 ± 8	NR	ORC/collagen matrix	Hydro-colloid dressing	VLUs
Motzkau et al., 2010 [15]	RCT	1	19	NR	NR	ORC/collagen matrix	Good standard wound care	DFUs
Ulrich et al., 2011 [28]	CCT	1	32	>18	22/10	ORC/collagen matrix	Hydro-colloid dressing	DFUs
Gottrup et al., 2013 [22]	RCT	2	39	NR	35/4	ORC/collagen/silver-ORC	Open wound healing	DFUs
Kloeters et al., 2015 [25]	RCT	1	33	>18	NR	ORC/collagen with foam dressing	Foam hydropolymer dressing	PIs
Cullen et al., 2017 [21]	RCT	3	49	24–90	31/18	ORC/collagen/silver-ORC	Standard of care	VLUs
Griffin et al., 2019 [23]	CCT	1	844	NR	NR	ORC/collagen/silver-ORC	Ovine (sheep-derived) collagen extracellular matrix	DFUs
Chowdhry, 2019 [20]	CRS	1	59	51.9 ± 14.4	27/32	ORC/collagen/silver-ORC	Petrolatum-based gauze dressing	Skin graft donor site wounds

Note: RCT, randomized clinical trial; CCT, comparative clinical trial; CRS, comparative retrospective study; ORC, oxidized regenerated cellulose; DFU, diabetic foot ulcer; VLU, venous leg ulcer; PI, pressure injuries; NR, not reported.

**Table 2:** Interventional characteristics of all included studies.

Authors	Type of wound	Wound duration	Wound area, test	Wound area, control	No. of test wounds	No. of control wounds	No. of dressing changes per week per patient, test	No. of dressing changes per week per patient, control	Follow-up
Veves et al., 2002 [29]	DFUs	<6 and >6 months	2.5 (0.2–27.4)	3.1 (0.1–42.4)	138	138	10.1	11.2	12 weeks
Vin et al., 2002 [30]	VLUs	NR	NR	NR	37	36	3.9 + 1.4 d	4.1 + 1.6 d	12 weeks
Lobmann et al., 2006 [26]	DFUs	NR	1237 mm sq	1132 mm sq	18	15	Daily	Daily	1 week
Luis Lazaro-Martinez et al., 2007 [27]	DFUs	NR	NR	NR	20	20	Every 2 days	Every 2 days	6 weeks
Kakagia et al., 2007 [24]	DFUs	≥3 months	25.8 ± 15.2	28.4 ± 13.6	17	17	NR	NR	8 weeks
Smeets et al., 2008 [13]	VLUs	NR	NR	NR	17	10	NR	NR	8 weeks
Motzkau et al., 2010 [15]	DFUs	NR	NR	NR	13	6	7	7	5 days
Ulrich et al., 2011 [28]	DFUs	NR	12 ± 6	14 ± 5	22	10	NR	NR	12 weeks
Gottrup et al., 2013 [22]	DFUs	NR	2.1 ± 3.1 cm sq	4.4 ± 6.3 cm sq	24	15	NR	NR	4 weeks
Kloeters et al., 2015 [25]	PIs	≥6 weeks	More than 1 cm sq	More than 1 cm sq	23	10	2–3 days	2–3 days	12 weeks
Cullen et al., 2017 [21]	VLUs	<12 and >12 months	6.9 ± 4.1	5.6 ± 3.0	22	27	Twice in a week	Twice in a week	12 weeks
Griffin et al., 2019 [23]	DFUs	NR	1.5 cm sq	1.5 cm sq	422	422	Once in 2 weeks	Once in 2 weeks	16 weeks
Chowdhry, 2019 [20]	Skin graft donor site wounds	NR	69.67 ± 9.45	69.13 ± 6.81	29	30	1.79 ± 0.73	0.67 ± 0.66	NR

Note: DFU, diabetic foot ulcer; VLU, venous leg ulcer; PI, pressure injury; NR, not reported.

RETRACTED

## Data Availability

The datasets used and/or analyzed during the current study are available from the corresponding author on reasonable request.
